# Using Artificial Intelligence Technology to Solve the Electronic Health Service by Processing the Online Case Information

**DOI:** 10.1155/2021/9637018

**Published:** 2021-11-26

**Authors:** Guoxiang Xu, Hao Jin

**Affiliations:** ^1^School of Statistics and Management, Shanghai University of Finance and Economics, Shanghai 200433, China; ^2^Research Center for Applied Statistics, Shanghai University of Finance and Economics, Shanghai 200433, China

## Abstract

With the continuous improvement of economic level and the continuous development of science and technology in China, information technology has begun to integrate into all walks of life. Medical units have begun to change from the traditional medical system to the intelligent system, and the processing of online case information has become an important component of medical informationization. To improve the efficiency of dealing with online case information, this study proposes to establish a fully connected neural network model to deal with online cases. Using jieba word segmentation tool and data preprocessing technology, the data of electronic medical records are sorted out, and the data are quantified using Word2Vec and other tools, and the data on electronic medical records are converted into one-hot binary variables. The quantified data are trained into a fully connected neural model, and the accuracy rate is about 88%. It is compared with naive Bayes and decision tree classification methods, and then a comparative experiment is carried out by solving e-health services in different ways. The results show that the fully connected neural network model has the best classification effect: the highest accuracy rate is about 93.7%, the highest precision rate is about 94.0%, the highest recall rate is about 95.3%, and the highest F1 score is about 94.6%. However, using artificial intelligence technology to solve electronic health services has great advantages, among which efficiency, assistance, and service satisfaction are all higher than 90%, which provides favorable technical support for electronic health services.

## 1. Introduction

Every country has some research on e-health services [1]. The United States introduced computers to assist calculation and then introduced the development and promotion of electronic medical record system. At the same time, Britain has also increased the research and development and promotion of electronic medical record system. Other countries are gradually developing their own electronic medical records to promote the informationization of medical services.

In the research field of electronic medical records, machine learning technology has been used to mine and extract data from electronic medical records [2, 3]. The commonly used machine learning methods are support vector model [4, 5], hidden Markov model, maximum entropy model [6], conditional random field model [7], etc. However, electronic medical records contain patient privacy information, which increases the difficulty of medical field corpus of electronic medical records [8]; at the same time, the medical professional background required by the corpus also limits its establishment [9]. Researchers conduct research on privacy removal of electronic medical records, patient status recognition, named entity recognition of electronic medical records, relationship extraction, etc., and organize relevant evaluation tasks to promote the development of related research [10]. In the evaluation task of named entity recognition in electronic medical records, the combination of conditional random fields and support vector machines has achieved good results, with 85.23%, 93.62%, and 73.13% in concept extraction, diagnosis detection, and relationship detection, respectively [11]. By extracting and encoding different entities, and counting the results of common occurrence of entities, the relationship between entities is identified; the precision rate is 92%, and the recall rate is 90% [12]. By constructing medical knowledge base, using bubble-bootstrapping method and relationship weight calculation method, we can realize the recognition of named entities and the extraction of entity relationships [13]. With the development of deep learning technology, deep learning models such as cyclic neural network and convolution neural network have been applied to natural language processing [14]. Whether it is the research of electronic medical record system or the data mining of electronic medical record using machine learning technology, the research of electronic medical record abroad, especially in English electronic medical record, is mature [15, 16], which is helpful to electronic health service.

In this study, the feasibility of the model is verified by establishing a fully connected neural network model for training; at the same time, it is compared with naive leaf bass and decision tree classification methods. At the same time, by adopting three ways, namely using artificial intelligence technology, not using artificial intelligence technology, and using other ways, we compare the efficiency, convenience, standard, and other indicators of dealing with online cases. Finally, the results show that artificial intelligence technology can effectively deal with online case information to solve the electronic health service. The second part of the study introduces the related knowledge of deep learning and data preprocessing technology. The third part analyzes the symptoms and diagnosis results in electronic medical records, and transforms and operates the data. In the fourth part, the fully connected neural network model in the deep learning model is explained and evaluated. In the fifth part, experiments are carried out under various models.

## 2. Related Technologies and Theories

### 2.1. Classification Method of Deep Learning Method

The application of deep learning method in classified tasks will improve work efficiency. For example, when the method of deep learning is applied to electronic cases, it can effectively assign the disease names on the cases to a category, which is convenient for doctors to read. The classification methods of deep learning include fully connected neural network and cyclic neural network. Compared with traditional machine learning methods, deep learning methods are quite different, and they can be effectively applied to speech recognition, text classification, image recognition, and other tasks.

### 2.2. Supervised Learning Theory

Supervised learning and unsupervised learning are the main learning tasks in the theoretical basis of machine learning and are the basis of artificial intelligence technology to deal with online cases.

Supervised learning is a marked learning task, and the common marked task is classification task. For classification, the input training data have characteristics and labels. Learning is to find the relationship between features and labels. When unknown data with features but without labels are input, the labels of unknown data are known through the existing relationships; that is, prediction is carried out according to new data. In the above classification, if all training data are labeled, it is supervised learning.

### 2.3. Data Preprocessing Techniques

#### 2.3.1. Word2Vec, A Natural Language Processing Tool

A natural language processing Word2Vec is a word vector tool, which is composed of two kinds of neural networks. By training the neural networks, the transformation of word vectorization can be realized. The relationship between words is mined by training, and then the cosine similarity is used to measure the distance between vectors. The closer the distance, the higher the similarity and relevance between words.

#### 2.3.2. Data Types of Binary Variables

Binary variable data types are implemented using vectors composed of 0 or 1. It is different from one-hot coded one-hot. There is only one 1 in one-hot coded vector, and the rest are all zeros. However, there are one or more ones in binary coded vector, which is very convenient to express symptom characteristics.

## 3. Data Preprocessing

### 3.1. Sources of Data

The data sources of this study include two aspects: the first is the online case data set of a 3A Hospital in Chongqing Province and the second is the online case data of Baidu Medical Encyclopedia.

Among them, the real patient case data come from a 3A Hospital in Chongqing Province, while Baidu Encyclopedia medical data are obtained by crawling, screening, and sorting its website through crawler, as shown in Table 1.

The scientific basis for determining the relationship between symptoms and diagnosis presented in Table 1 is based on the summary of symptoms presented by patients on medical records and diagnosis given by doctors. The judgment of targeted medical effect has a certain scientific judgment basis.

### 3.2. Data Processing

The purpose of data processing is to transform messy medical data into a format that can be recognized and processed by computers or machine learning models. Chinese word segmentation tool jieba is used to segment the descriptive symptoms on electronic cases, and the descriptive symptom nouns are accurately separated and extracted, but jieba word segmentation tool has some disadvantages, such as limited recognition of symptom nouns, inability to segment symptom nouns accurately, and inability to judge the symptom attributes of words. To solve these problems, the following improvements have been made:

First, using loading dictionary, the collected disease and symptom nouns are sorted and summarized, and the dictionary is made using jieba word segmentation tool and loaded into jieba word segmentation. By scanning the vocabulary of trie tree structure, the symptom nouns are imported into trie tree. Trie tree means that the first few words of words are the same, which is convenient for trie tree storage and improves the search speed.

Second, for dictionary supplement, to accurately segment some positive symptoms, “negative” symptom descriptions to the dictionary are added, as shown in Table 2, and jieba tool of symptom noun dictionary is loaded. In the screening of nouns describing symptoms, the nonexistent words are removed and the words in the symptom dictionary are retained. The final effect is shown in Table 3. For diagnostic data segmentation, to extract the disease name after word segmentation, the original disease with disease name is replaced, the words after word segmentation are screened first, the words in the existing and diagnostic dictionary are kept, and the words that do not exist are deleted. Effective screening is implemented by the rules in Table 4.

### 3.3. Data Conversion

#### 3.3.1. Symptom Data Transformation

Each visit of the patient is recorded as a sample, and multiple symptoms will appear in the symptom description, because each sample is represented by 0 and 1 vectors, as shown in Table 5.

#### 3.3.2. Diagnostic Data Transformation

Each patient's visit record is taken as each sample, and there will only be one diagnosis result in each diagnostic data, with a total of 1277 symptoms. The data are converted by one-hot, as shown in Table 6.

Finally, the total number of samples is 22176, while the disease symptoms with characteristics can be converted into 1227 data types and the disease diagnosis can be converted into 2018 one-hot data types.

## 4. Deep Learning Model

The above processed data are trained using the following fully connected neural network.

### 4.1. Fully Connected Neural Network

There are 1227 neurons in the input layer of the fully connected neural network, and there are 1227 disease symptoms accordingly; there are 2018 neurons in the output layer, and there are 2018 diseases accordingly. The model can input 1227 symptoms and diagnose 2018 disease types. However, the sample data are sparse, with 2048 neurons in the first hidden layer and 1024 neurons in the second hidden layer, as shown in Figure 1.

In this study, we use the neural network model, through the forward propagation method combined with data preprocessing, and obtain the forward propagation formula of the input layer as follows:

(1) fx=ReLU∑kn=1227XkWk±b.

In formula (1), *n* corresponds to 1227 disease symptoms, *X* represents each symptom, and *W* represents the weight of each symptom, and then, multiplying and adding the total symptoms and the corresponding weights, *b* represents the bias value in the formula, and the calculated structure is represented by the function ReLU for nonlinear changes. The schematic diagram of ReLU is shown in Figure 2.

The automatic weight adjustment method of fully connected neural network uses back-propagation technology. Through the input symptom vector, it propagates forward to the output layer, compares the output result of the output layer with the real diagnosis result, and calculates the error between them by the following formula:

(2) $$\begin{array}{c} E\left(f\left(x\right),y\right)=-\sum_{k}^{n=1227}y_{k}\log\left(f\left(x\right)\right). \end{array}$$

The calculation of error is the operation between the vector points and the addition. When there are 2018 neurons in the output layer, 2018 diseases are predicted, and then, the prediction probability of 2018 diseases is output using forward propagation. Then, through the error calculation with 2018 diagnostic vectors, the error value is brought to the output layer, and the weight value is updated, which is expressed by the following formula:

(3) $$\begin{array}{c} \frac{\partial E_{total}}{\partial W_{layer2}}=\frac{\partial E_{total}}{\partial O}*\frac{\partial O}{\partial L_{2}}*\frac{\partial L_{2}}{\partial W_{layer2}}. \end{array}$$

In the formula, *W*_*layer*2_ represents the updated weight and then *E*_*total*_ represents the error between the predicted value and the true value, and the weight is updated in the negative direction. The formula is as follows:

(4) $$\begin{array}{c} W_{layer2}=W_{layer2}-\frac{\partial E_{total}}{\partial W_{layer2}}. \end{array}$$

#### 4.1.1. Activation Function

The activation function ReLU is used between the hidden layers, as shown in Figure 3. Its advantage is to make the update effect better and prevent the gradient from disappearing during the update process to the greatest extent. The formula is as follows:

(5) ReLUz=max0,z.

The activation function Softmax is used between the output layers, as shown in Figure 4. Its function is to classify various diseases and predict the probability of diseases. The formula is as follows:

(6) $$\begin{array}{c} S_{i}=\frac{e^{i}}{\sum {}_{j}e^{j}}. \end{array}$$

#### 4.1.2. Optimization

In the dropout layer, neurons are randomly selected, which is the Bernoulli distribution. A certain probability is randomly selected between 0 and 1, to inactivate the current neural network neurons and prevent overfitting and normalization. The neural network model uses a dropout value of 0.5, and each prediction retains 50% of the hidden layer neurons. The forward propagation formula after using dropout is as follows:

(7) $$\begin{array}{c} r_{j}^{1}∼Bernoulli\left(p\right),\\ x^{l}=r^{l}*y^{l},\\ z^{\left(l+1\right)}=W_{i}^{l+1}x^{l}+b_{i}^{l+1},\\ y_{i}^{l+1}=f\left(z_{i}^{l+1}\right), \end{array}$$

where *r* is the random inactivation rate, which obeys Bernard's distribution, the best *R* is determined by grid search and comparison training curve, as shown in Figure 5.

#### 4.1.3. Number of Iterations

There are 15 iterations in this model. It can be concluded from the figure that the number of iterations is directly proportional to the accuracy rate. When the number of iterations is 15, the accuracy rate is 87%. To prevent overfitting, the number of iterations is 15, as shown in Figure 6.

#### 4.1.4. Evaluation Function

top_k_compliance as the evaluation function is used. K stands for accuracy, which means that the real sample is in the first K bits of the prediction probability, that is, the correct prediction. In this study, the K value is 10. If there are real samples in the top 10 predicted diseases, it means correct prediction.

#### 4.1.5. Parameter Optimization Algorithm

The gradient descent algorithm Adam is used to optimize the parameters by back propagation.

### 4.2. Model Evaluation

The parameter settings of the fully connected neural network model are shown in Table 7.

The total data of 22176 are divided into three parts, which are training data set, verification data set, and test data set. Their ratio is 18 : 1: 1, and the evaluation function is top_k_accessibility (*k* = 10). The final model experimental results are shown in Table 8, while the training convergence diagram of fully connected neural network is shown in Figure 7.

### 4.3. Model Problem Analysis

As can be seen from convergence Figure 7, the model has a fitting phenomenon, with a training error of about 99%, but a test error of about 87%. The reason is that the data are unevenly distributed, and the number of diseases in different samples is different. For example, common cold symptoms such as upper respiratory tract infection and acute pharyngitis account for the majority of the samples, while diseases such as heart disease account for a small part, as shown in Figures 8 and 9.

Due to the complexity of the model, there are 2018 diseases in the data, but the sample size is 22,176. Because the number of samples is too low and the number is too small, it is easy to overfit.

## 5. Experimental Results and Analysis

### 5.1. Evaluation Indicators

The fully connected neural network is one of the classification methods in deep learning, which usually uses accuracy, precision, recall, and F_1_ scores in classification tasks. Combined with the forecast and actual situation during classification, the correct rate, precision rate, recall rate, and F1 value are calculated by the following formulas:

(8) $$\begin{array}{c} \text{Accuracy}=\frac{TP+TN}{TP+FP+TN+FN},\\ \text{Precision}=\frac{TP}{TP+FP},\\ \text{Recall}=\frac{TP}{TP+FN},\\ F_{1}=\frac{2\times \text{Precision}\times \text{Recall}}{\text{Precision}+\text{Recall}}. \end{array}$$

At the same time, this experiment also uses artificial intelligence technology, other methods, and methods without artificial intelligence technology to deal with online cases, and in solving electronic health services, their efficiency, assistance, service satisfaction, and other indicators.

### 5.2. Experimental Results

The experimental results under different classification methods are shown in Table 9.

It can be seen from the data in Table 9 that the fully connected neural network has achieved excellent results compared with other methods in this experiment. The highest accuracy rate can reach 93.7%, the highest precision rate can reach 94%, the highest recall rate can reach 95.3%, and the highest F1 score can reach 94.6%. Compared with the other four classification methods, the classification method of fully connected neural network has achieved the highest effect on the treatment of online cases.

Three methods are adopted, namely using artificial intelligence technology (A), not using artificial intelligence technology (B), and using other methods (C), in solving electronic health services, such as efficiency, convenience, standard, assistance to doctors, and user satisfaction with its services. The experimental results are shown in Table 10.

It can be seen from the data in Table 10 that Mode A (using artificial intelligence technology) can effectively solve the problem of electronic health service. Compared with the other two methods, it is the best. In this experiment, Mode A has the highest efficiency of 98% in solving electronic health services, 92% in doctor assistance, 94% in convenience, 96% in data standard, and 96% in service satisfaction.

### 5.3. Analysis of Experimental Results

According to the experimental results of the above different classification methods, the results are compared and analyzed. The accuracy, precision, recall, and F1 scores of the data under different classification methods are shown in Figures 10–13, respectively.

As can be seen from the figure, when the classification method of fully connected neural network classifies different data of online cases, the accuracy, precision, recall, and F1 scores are all higher than those of the other four classification methods (naive Bayes, decision tree, support vector machine, and logistic regression), and their maximum values are all more than 93%, which fully demonstrates the superiority of fully connected neural network in online case information processing.

According to the experimental results of different modes in Table 10, the results are analyzed. We should adopt different ways to deal with online cases, from the efficiency, assistance, standardization, and convenience of treatment, so as to improve the service satisfaction of electronic health services as shown Figure 14.

It can be seen from the figure that only Mode A (using artificial intelligence technology) is significantly higher than the other two ways in efficiency, assistance, convenience, standard, and service satisfaction. Therefore, we know that artificial intelligence technology works best in solving electronic health services. The future work focuses on the problem of small sample size of electronic medical records and deeply analyzes the feasibility of electronic medical record statistics under large data volume. Through the continuous study of the scientific nature between disease and diagnosis on samples, further analysis is needed, and decision analysis is carried out under a large number of case samples and clinical trials.

## 6. Conclusion

In conclusion, this study constructs a model based on the fully connected neural network and trains the processed data to verify the feasibility of the model. The results show that the verification accuracy and the test accuracy of the fully connected neural network model are 88.25% and 88.81%, respectively. Compared with different classification methods, the accuracy and precision of different data classification methods are compared. At the same time, by adopting three ways, namely using artificial intelligence technology (A), not using artificial intelligence technology (B), and using other ways (C), we compare the efficiency, convenience, standard, and other indicators of dealing with online cases.

According to the comparison results of different experiments, the fully connected neural network model has the highest efficiency in processing electronic medical records, and the indicators of electronic health services have been greatly improved by using artificial intelligence technology to deal with electronic health services.

However, there are still the following problems to be further studied in this study. On the one hand, due to the uneven distribution of selected data and the number of diseases in different samples, the fully connected neural network model has fitting phenomenon. On the other hand, the indicators selected in this study cannot be fully covered, and the selected indicators cannot fully reflect the analysis value. All these need to be further studied and improved in the future.

## Figures and Tables

**Figure 1:** Structural diagram of fully connected neural network.

**Figure 2:** Schematic diagram of ReLU.

**Figure 3:** ReLU activation function.

**Figure 4:** Softmax activation function.

**Figure 5:** Dropout and top_k_acquisition training curves.

**Figure 6:** Training curves of epoch number and top_k_accessibility.

**Figure 7:** Training convergence diagram of fully connected neural network.

**Figure 8:** Number of disease occurrences in the sample.

**Figure 9:** Number of low-frequency diseases.

**Figure 10:** Comparison of accuracy rates of five methods.

**Figure 11:** Comparison of precision ratio of five methods.

**Figure 12:** Comparison of recall rates of five methods.

**Figure 13:** Comparison of F1 scores of five methods.

**Figure 14:** Comparison under different modes. (a) Type 1 comparison results. (b) Type 2 comparison results. (c) Type 3 comparison results.

**Table 1:** Original data.

Symptom	Diagnose
The patient developed fever, sore throat, cough, and no cough 2 days ago. No nasal congestion, runny nose, chest tightness, pneumatic foot, nausea, vomiting, abdominal pain, abdominal distension, and urgency and pain in urination, so he came to our hospital for treatment.	Fever cause: acute pharyngeal bronchitis

Two days ago, the patient appeared dizziness, unconscious disorder, no nausea, vomiting, chest tightness, shortness of breath, no speech disorders, no abdominal pain, abdominal distension, and no limited limb movement, so he came to our hospital for treatment.	Causes of dizziness: coronary heart disease due to cerebral ischemia

**Table 2:** Supplement to symptom dictionary.

Original symptom	Negative symptom
Polyuria	No polyuria
Fever	No fever
Sore throat	No sore throat

**Table 3:** Screening of word segmentation results.

Original symptom description	Screening results of word segmentation symptoms
The patient developed fever, sore throat, cough, and no cough 2 days ago. No nasal congestion, runny nose, chest tightness, pneumatic foot, nausea, vomiting, abdominal pain, abdominal distension, and urgency and pain in urination, so he came to our hospital for treatment.	Sore throat, fever, runny nose, cough, no urgency, no nasal congestion, no expectoration, vomiting, no abdominal pain, no nausea, abdominal distension, no chest tightness, and pain in urine.

Two days ago, the patient appeared dizziness, unconscious disorder, no nausea, vomiting, chest tightness, shortness of breath, no speech disorders, no abdominal pain, abdominal distension, and no limited limb movement, so he came to our hospital for treatment.	No speech disorder, unconscious disorder, vomiting, no abdominal pain, no nausea, dizziness, abdominal distension, and no chest tightness.

Five hours ago, the patient developed dizziness, accompanied by line of sight rotation, nausea, vomiting of stomach contents, unconscious disorder, no chest tightness, shortness of breath, no abdominal pain, abdominal distension, no speech disorders, and no limited limb movement. He came to our hospital for treatment and asked for infusion treatment.	No speech disorder, no unconscious disorder, no abdominal pain, vomiting, stomach contents, dizziness, abdominal distension, no chest tightness, and nausea.

**Table 4:** Screening of diagnostic word segmentation rules.

Original diagnosis result	Rule filter results	Screening rule
Hypertension grade 3 and high risk	Hypertension	Removal of disease level
Type 2 diabetes mellitus	Diabetes mellitus	Detailed types of diseases removed
Bronchitis chronic bronchitis	Chronic bronchitis	Keeping the most detailed disease name

**Table 5:** Symptom data transformation 0 and 1 vectors.

Sample	Symptom	Coughing	Runny nose	Fever	Nasal obstruction
Patient 1	Cough and stuffy nose	1	0	0	1
Patient 2	Fever cough	1	0	1	0
Patient 3	Fever due to nasal obstruction	0	0	1	1

**Table 6:** Diagnostic data.

Sample	Diagnose	Gastritis	Bronchitis	Cold
Patient 1	Gastritis	1	0	0
Patient 2	Bronchitis	0	1	0
Patient 3	Cold	0	0	1

**Table 7:** Model parameter setting of fully connected neural network.

Input layer	Dropout	Evaluation function	Parameter optimization algorithm
(22176, 1227)	0.5	top_k_accuracy	Adam

**Table 8:** Experimental results.

Model	Accuracy	
	Verification accuracy (%)	Test accuracy (%)
Fully connected neural network	88.25	88.81

**Table 9:** Experimental results under different classification methods and different indexes (%).

Classification method	Different data	Correct rate	Precision	Recall rate	F_1_ score
Naive Ye Besi	Data A	42.8	46.1	47.9	47.0
	Data B	44.3	45.9	48.5	47.2
	Data C	45.1	46.1	46.7	47.3
	Data D	51.6	55.1	53.0	54.0

Decision tree	Data A	72.5	71.9	72.9	72.4
	Data B	71.2	73.8	72.3	73.0
	Data C	73.1	74.2	73.2	74.1
	Data D	75.6	74.7	75.9	75.3

Support vector machine	Data A	73.6	75.1	73.4	74.2
	Data B	64.9	65.5	74.1	69.5
	Data C	64.1	64.5	65.3	65.2
	Data D	65.1	64.1	76.0	69.5

Logistic regression	Data A	53.7	49.9	78.6	61.0
	Data B	47.3	49.5	56.0	52.5
	Data C	46.4	45.6	48.1	47.2
	Data D	48.2	51.6	59.9	55.4

Fully connected neural network	Data A	76.8	77.9	80.6	82.4
	Data B	85.6	86.7	85.9	85.3
	Data C	88.1	88.8	89.1	89.3
	Data D	93.7	94.0	95.3	94.6

**Table 10:** Experimental results of different methods (%).

Type	Mode	Efficiency	Auxiliary degree	Convenience	Standard degree	Service satisfaction
Type 1	A	98	91	86	96	90
	B	45	21	31	23	37
	C	67	51	67	49	53

Type 2	A	95	89	93	93	96
	B	56	12	39	13	32
	C	71	45	69	58	45

Type 3	A	91	92	94	91	89
	B	31	13	41	27	41
	C	64	48	78	54	59

## Data Availability

The experimental data used to support the findings of this study are available from the corresponding author upon request.
